The article "Clinical Research on Gastrointestinal Surgery Based on Smart Medicine" was retracted in 2022. Reason: concerns about the peer review.

# Clinical Research on Gastrointestinal Surgery Based on Smart Medicine

**DOI:** 10.1155/2022/3698721

**Published:** 2022-03-21

**Authors:** Yang Lu

**Affiliations:** The Fourth Clinical Medical College, Zhejiang Chinese Medical University, Hangzhou 310000, Zhejiang, China

## Abstract

Smart medical technology uses the medical information platform, with the help of current technical means, so that the information between medical staff and medical equipment can be shared. The combination of current technology and the medical field has become the norm. In the future, more artificial intelligence technologies will be incorporated in the medical field to promote the development of medical undertakings. At present, the information on the Internet is very large and complex, and general search engines often do not have knowledge in certain professional fields and can only perform shallow keyword searches, so it is difficult to meet people's medical diagnostic needs. Smart medical technology can solve the problem of these needs. Surgery, commonly known as operation, refers to the process of entering the body to change the condition of the disease through technical means and under the guidance of professionals. Earlier operations only performed cutting on the body surface. With the continuous maturity of surgical operations, operations can now be performed on any part, but manual operations are still the main one. In addition to manual surgery, there are many machine surgeries, such as laser surgeries. Clinical research takes the diagnosis and treatment of diseases as the main content, takes patients as the research object, and is a scientific research activity involving multiple personnel. This article aimed to study the clinical research of gastrointestinal surgery based on smart medicine and hoped to use smart medical technology to improve the clinical research level of gastrointestinal surgery and provide technical support for surgery. This study proposes to apply natural language processing technology to the medical field, build an intelligent diagnostic auxiliary system, and use the existing medical record data to realize the corresponding medical auxiliary function. The research measures and analyzes the basic information of medical students, the incidence of functional gastrointestinal disease, the incidence of common symptoms of functional gastrointestinal disease, and the differential distribution of various symptoms in different professions, genders, and ages. The experimental results of this article show that there are 27 cases of gastrointestinal bleeding, accounting for 18%; 10 cases of dysphagia, accounting for 7%; 78 cases of abdominal pain and bloating, accounting for 53%; and 19 cases of melena, accounting for 13%. Abdominal pain and bloating are the most common clinical manifestations of the gastrointestinal tract and require more attention.

The article "Clinical Research on Gastrointestinal Surgery Based on Smart Medicine" was retracted in 2022. Reason: concerns about the peer review.

## 1. Introduction

With the improvement of living standards, the average life expectancy of people has begun to extend, the birth rate of the population has been declining, and people are paying more and more attention to health. The demand for medical treatment began to increase, leading to a shortage of medical resources in the society and a shortage of medical staff. How to optimize the allocation of resources based on the limited medical resources, improve the utilization rate of medical resources, and alleviate the contradiction between doctors and patients is a problem that needs to be solved urgently. In addition to the shortage of medical resources, the contradiction between doctors and patients may also be due to the lack of smooth channels for rights protection, or the accident caused by the patient's own reasons. In addition, changes in the environment have led to various intractable diseases, and the monitoring of these diseases needs to be rigorous. For example, the composition of crustal materials in life will have different effects on human health, and iodine deficiency can lead to endemic goiter. Based on this situation, intelligent medical treatment has emerged. The system monitors the patient's blood pressure and body temperature, so that users can inquire about relevant conditions in time, which saves medical resources to a certain extent. Patients can also communicate directly with doctors through smart medical equipment to improve treatment efficiency. Gastrointestinal surgery is a relatively common operation, but functional gastrointestinal diseases have complex conditions and slow treatment effects and may be accompanied by complications after the operation. Therefore, combining smart medical methods with gastrointestinal surgery, it is expected that smart medical technology can improve treatment efficiency, alleviate complications, and promote the progress of related medical fields.

The use of intelligent medical systems to integrate cases can realize the medical assistance of cases, improve the efficiency and effectiveness of diagnosis, promote the scientification of clinical medical treatment, and avoid diagnostic accidents caused by personal errors of medical staff. Due to the differences in personal medical knowledge and experience, each doctor has different medical records. By categorizing different medical records, the format of the medical records can be standardized, which facilitates the sharing of information among medical staff. The intelligent medical system can reduce the workload of medical staff and relieve the pressure of medical staff [1, 2].

The article "Clinical Research on Gastrointestinal Surgery Based on Smart Medicine" was retracted in 2022. Reason: concerns about the peer review.

As the main body of society, “people” pay the most attention to people. The current living conditions are improving day by day, and people are paying more and more attention to health, which leads to a shortage of medical resources. How to alleviate the contradiction in medical resources is a hot topic at the moment. Büyükzkan and Ger proposed a new method for evaluating the selection process of smart medical equipment in a group decision-making environment in an uncertain decision-making environment. The intuitionistic fuzzy integral method is used to deal with the uncertainty and ambiguity in the decision-making process. The method also considers the interaction between the decision criteria in the data provided by the decision-maker. He focused on the wearable monitoring devices chosen by heart patients. It is hoped to arouse the interest of experts in the healthcare industry through complex issues and evaluate smart medical devices according to different evaluation criteria [3]. With the development of information technology, the concept of smart medical care has gradually emerged. Smart health care utilizes new-generation information technologies such as the Internet of things, big data, cloud computing, and artificial intelligence to comprehensively transform the traditional medical system, making medical treatment more efficient, convenient, and personalized. To introduce the concept of smart medicine, Tian et al. first listed the key technologies that support smart medicine, introduced the current status of smart medicine in several important areas, then elaborated on the existing problems of smart medical care, and tried to propose solutions [4]. Ronen et al. examined whether men's and women's autonomous response patterns to pain (defined as increased heart rate and blood pressure) were different during the entire anesthetized abdominal surgery and collected baseline blood pressure and heart rate data, and blood pressure and heart rate measurements after the surgical incision. The baseline data and postoperative incision data were compared to assess whether the blood pressure and heart rate change patterns of men and women are different, and it was found that women had a stronger pain response [5]. Hill et al. studied 333 hospitalized patients who were discharged home after weight loss, benign foregut, liver, pancreas, abdominal hernia, and colon surgery. Chronic opioid users or patients with complications were excluded. Through questionnaires and telephone surveys, the patients' family opioid use was quantified, and it was found that 85% of patients took opioids. 15 opioids met 88% of the opioid needs of patients discharged from the hospital on the first postoperative day. A multivariate analysis of patients discharged after the first day showed that the number of opioids used at home was related to the number of opioids taken the day before discharge, but was not related to the type of surgery [6]. Kafalä et al. evaluated the weight loss, metabolic parameters, and postoperative complications of patients undergoing laparoscopic gastric bypass and laparoscopic sleeve gastrectomy. By comparing the patient's age, gender, body mass index, operation time, surgical complications, hospital stay, and long-term follow-up results, it was found that during the study period, 91 patients (45 cases of laparoscopic Roux-en-Y gastric bypass and 46 cases of laparoscopic sleeve gastrectomy) underwent bariatric surgery. There was no difference between the two groups in terms of preoperative patient characteristics. Compared with preoperatively, both groups showed statistically significant weight loss and improvement in complications [7]. Studying new models of the intestine is the key to understanding intestinal diseases and developing new therapies. The intestinal organ-like culture system has greatly promoted the research of human gastrointestinal tract. Blutt et al. explored how organs and intestinal cultures become biological and physiological related systems to study the impact of symbiotic organisms and the pathogenesis of human infectious diseases. These cultures can be established from many donors, and they retain the genetic and biological characteristics of the donor. This experiment can discover host-specific factors that affect susceptibility to infection and develop personalized treatment methods [8]. Ho et al. focused on the three fatty acid-binding proteins found in the gastrointestinal tract and discussed their role as diagnostic or disease monitoring markers in neonatal necrotizing enterocolitis, acute mesenteric ischemia, celiac disease, and inflammatory bowel disease. Among the three fatty acid-binding proteins, intestinal fatty acid-binding proteins have received the most attention. Regardless of the underlying cause, the increase in intestinal fatty acid-binding protein in blood and urine reflects intestinal cell damage. The short half-life of intestinal fatty acid-binding protein also means that it is a relatively sensitive marker. In contrast, there is currently little evidence to support liver fatty acid-binding protein and ileal bile acid-binding protein as sensitive biomarkers under these conditions [9]. Although these theories have discussed smart medicine, extra-GI surgery, and clinical research to a certain extent, the content of the discussion only revolves around a part and does not combine the three, so it is not practical.

The article "Clinical Research on Gastrointestinal Surgery Based on Smart Medicine" was retracted in 2022. Reason: concerns about the peer review.

This study proposes for the first time to standardize business processes in a smart medical environment, simulate the randomness of the environment and the concurrency of the process after the introduction of smart medical equipment and systems, and improve the efficiency of the actual work process. After the operation, the complications of gastrointestinal surgery are discussed, and the patient's postoperative recovery is evaluated.

## 2. Clinical Research Methods Based on Smart Medicine in Gastrointestinal Surgery

### 2.1. Smart Medical Technology

Smart medical technology originated in the United States, and developed countries began to explore it in the early part of the last century [10, 11]. The intelligent medical system was initially applied in hospitals, but it did not develop a wide range of applications, mainly to detect the body of the patient, and then transmit specific data to the doctor, and the doctor makes judgment and analysis based on the data [12]. The initial smart medical structure is shown in Figure 1.

With the continuous popularization of computer technology and the Internet, it is inevitable to integrate it with the medical field. In this context, smart medical care has also developed rapidly [13, 14]. Traditional smart medical care only appears in hospitals, but now smart medical care has become popular, and it has been able to provide personalized services. The widespread wearable medical equipment is the result of smart medical care [15, 16]. The device monitors the patient's physical condition and sends messages to family members and nearby hospitals in case of unhealthy conditions, saving rescue time. Patients can also query their own physical data at any time to understand their own condition in time [17]. The system structure is shown in Figure 2.

Through continuous improvement, intelligent medical technology can make reasonable diagnosis through the computer technology in its own system [18, 19]. Smart medical technology can summarize existing medical knowledge and experience to form a data inventory into the system, then analyze according to the patient's various data, make simple judgments, and provide certain suggestions to the doctor. The system can make inferences based on the patient's clinical manifestations and age and gender combined with the database. Although there are deficiencies, this is a major breakthrough in the intelligent system [20, 21]. The intelligent diagnostic system is shown in Figure 3.

### 2.2. Classification Technology

A principal component analysis is a different statistical technique based on dimensionality reduction methods. The main principle is to organize disordered data into an ordered data set [22].

(1) $$\begin{array}{c} Q_{ab}=\frac{s_{ab}-{\bar{s}}_{b}}{s_{b}},a=1,2,\ldots g,b=1,2,\ldots k. \end{array}$$

Here,

(2) $$\begin{array}{c} {\bar{s}}_{b}=\frac{\sum_{a}^{g}s_{ab}}{g},\\ L_{b}^{2}=\frac{\sum_{a}^{g}\left(s_{ab}-{\bar{s}}_{b}\right)}{g-2}. \end{array}$$

Formula (1) is a function expression for data standardization.

The article "Clinical Research on Gastrointestinal Surgery Based on Smart Medicine" was retracted in 2022. Reason: concerns about the peer review.

When calculating the incidence matrix of the formula, it can be expressed as follows:

(3) $$\begin{array}{c} W={\left(w_{ab}\right)}_{h}sh=\frac{m^{d}m}{g-2}. \end{array}$$

Here,

(4) $$\begin{array}{c} w_{ab}=\frac{\sum m_{db}m_{db}}{g-2},a,b=1,2,\ldots ,g. \end{array}$$

When the components of the matrix are determined:

(5) $$\begin{array}{c} \left|W-\varphi f_{h}\right|=0,\frac{\sum_{b}^{g}\varphi_{b}}{\sum_{b}^{q}\varphi_{b}}\geq 0.74. \end{array}$$

Solving formula (5), the value of *g* can be determined.

(6) $$\begin{array}{c} V_{ab}=m_{a}^{F}l_{b}^{c},b=1,2,\ldots ,g. \end{array}$$

Here, *V* represents the target component, so we can assume that *V*_*g*_ is the *g*th component.

(7) $$\begin{array}{c} O=\left(\left(a_{1},b_{1}\right),\left(a_{2},b_{2}\right),\ldots ,\left(a_{j},b_{j}\right)\right). \end{array}$$

Here, a represents the input space, *b* ∈ (−2,2).

(8) $$\begin{array}{c} u\left(a\right)=\mathrm{sgn}\left(h\left(a\right)\right). \end{array}$$

*u*(*a*) means *a* is a real value, and *b* > 0 at this time.

(9) $$\begin{array}{c} conv\left(D\right)=\left(a=\sum_{k}^{s}\alpha_{k}a_{k}|\sum_{k}^{s}\alpha_{k}=2\right). \end{array}$$

Here, *a*, *b*=2, *α*_*k*_ ≥ 0, and *k*=1.

(10) $$\begin{array}{c} conv\left(d\right)=\left(a=\sum_{k}^{s}\alpha_{k}a_{k}|\sum_{k}^{s}\alpha_{k}=2\right). \end{array}$$

Here, *a*, *b*=−2, *α*_*k*_ ≥ 0, and *k*=1.

Formulas (9) and (10) are shown in Figure 4.


(11) $$\begin{array}{c} a=\sum_{k}^{s}\beta_{k}a_{k}, \end{array}$$

(12) $$\begin{array}{c} a^{\prime }=\sum_{k}^{s}\beta_{k}a_{k}^{\prime }. \end{array}$$

Formula (11) represents the set point of the positive class, and formula (12) represents the set point of the negative class.

(13) $$\begin{array}{c} \left(\gamma *a\right)+l=\left(\gamma *\sum_{k}^{s}\beta_{k}a_{k}\right)+l=\sum_{k}^{s}\beta_{k}\left(\left(\gamma *a_{k}\right)+l\right), \end{array}$$

(14) $$\begin{array}{c} \left(\gamma *a^{\prime }\right)+l=\left(\gamma *\sum_{k}^{s}\beta_{k}a_{k}^{\prime }\right)+l=\sum_{k}^{s}\beta_{k}\left(\left(\gamma *a_{k}^{\prime }\right)+l\right). \end{array}$$

Among them, formula (13) is greater than zero, and formula (14) is less than zero.

(15) $$\begin{array}{c} \left(\gamma *a\right)+l\geq \varpi ,\\ \left(\gamma *a^{\prime }\right)+l\leq -\varpi . \end{array}$$

Here, (*γ∗a*)+*l*=0, and *ϖ* > 0.

(16) $$\begin{array}{c} u_{k}\left[\left(\gamma *a_{k}\right)+l\right]\geq 0,k=1,2,\ldots ,j, \end{array}$$

(17) $$\begin{array}{c} \underset{k=1,2,\ldots ,j}{\min}|\left(\gamma *a_{k}\right)+l|=2. \end{array}$$

Formula (16) represents the expression of hyperplane function. A hyperplane can be obtained by multiplying (*γ*, *l*) with any nonzero number. When the condition of formula (17) is satisfied, the plane is also called a normal hyperplane.

(18) $$\begin{array}{c} \left(\gamma *a_{k}\right)+l\geq 2,u_{k}=2, \end{array}$$

(19) $$\begin{array}{c} \left(\gamma *a_{k}\right)+l\leq -2,u_{k}=-2. \end{array}$$

When the sample set satisfies the conditions of formula (18) and formula (19), there is a unique canonical hyperplane.

The article "Clinical Research on Gastrointestinal Surgery Based on Smart Medicine" was retracted in 2022. Reason: concerns about the peer review.

### 2.3. Clinical Surgery

Clinic refers to the behavior of directly contacting the patient and observing the patient at close range [23]. All operations involved in this article refer to surgical operations. Surgery is the process of transforming the structure of the body by entering the human body with external force. Surgery is also a process of continuous development and evolution. Earlier surgery was just suture on the body surface, so it is popular to say that early surgery is the incision and suture of the tissue [24, 25]. With the continuous popularization of technology, current surgical operations can be performed on any part of the body with the help of technical means, even without too much cutting. When it comes to surgery, we have to talk about disinfection. The process of disinfection is very important to surgery and can greatly reduce the mortality rate of surgery. Usually, the disinfection process is carried out before the operation, and the purpose is to prevent bacterial infections around the operation, causing problems in postoperative recovery [26, 27]. Common disinfection methods include antibacterial and sterilization methods, which are introduced with the doctor wearing the surgical method as an example. The method of wearing a sterile surgical gown is to gently shake the surgical gown open, lift both sides of the collar, insert the hands into the sleeves, and stretch arms forward. After the itinerant nurse assisted in putting it on, the belt was lifted with arms crossed and sent to the back, and the nurse tied it behind him. The doctor did not need to touch the protective clothing with the disinfected hands to avoid contamination.  Figure 5 shows the whole process of the operating room:

## 3. Clinical Research Experiment Based on Smart Medicine in Gastrointestinal Surgery

### 3.1. Subjects

In this experiment, to explore the clinical situation of gastrointestinal surgery, we conducted a survey of gastrointestinal patients in city A during a certain period of time. Among the subjects surveyed, only gastrointestinal diseases are involved, which avoids the influence of other causes on the experiment.

The article "Clinical Research on Gastrointestinal Surgery Based on Smart Medicine" was retracted in 2022. Reason: concerns about the peer review.

According to the data in Table 1, this experiment surveyed 148 patients, 83 male patients and 65 female patients. In terms of the composition of male and female patients, male patients accounted for 56.1% and female patients accounted for 43.9%, and the proportion of men suffering from gastrointestinal tract was slightly higher than that of women. There were 3 patients aged 0–20, 30 patients aged 21–40, 44 patients aged 41–60, and 71 patients aged 60–80. According to the age of illness, the greater the probability of gastrointestinal disease with increasing age, especially in people over 60 years of age, the disease is more common.

### 3.2. Clinical Manifestations

Clinical manifestations in medicine refer to the symptoms of fever and weakness that occur after a patient suffers from a certain disease. There are many clinical manifestations of gastrointestinal disease, and the specific conditions are as follows.

According to the data in Table 2, the clinical manifestations of gastrointestinal diseases include gastrointestinal bleeding and abdominal pain and bloating. According to the survey, there were 27 cases of gastrointestinal bleeding in this experiment, accounting for 18%; 10 cases of dysphagia, accounting for 7%; 78 cases of abdominal pain and bloating, accounting for 53%; 19 cases of melena, accounting for 13%; and 14 cases of other clinical symptoms, accounting for 9%. According to the data, abdominal pain and bloating are the most common gastrointestinal clinical manifestations, followed by gastrointestinal bleeding and melena symptoms.

### 3.3. Location of Disease

There are many causes of gastrointestinal disease, which may be caused by problems in the uterus or problems in the stomach. The specific conditions are as follows.

According to the data in Table 3, there are many sites that cause gastrointestinal diseases. According to survey data, there are 3 cases that require surgery for ovarian reasons, accounting for 2%, and 19 cases that require surgery for colorectal reasons, accounting for 13%. There were 7 cases that needed surgery for peritoneal reasons, accounting for 5%, and 2 cases that needed operation for uterine reasons, accounting for 1%. There were 96 cases requiring surgery for gastric reasons, accounting for 65%, and 21 cases requiring surgery for duodenal reasons, accounting for 14%. According to the data, it can be seen that the most cases of surgery are due to stomach reasons, followed by the duodenum and colorectum, and the least cases of surgery are due to uterine reasons.

The article "Clinical Research on Gastrointestinal Surgery Based on Smart Medicine" was retracted in 2022. Reason: concerns about the peer review.

According to the data in Table 4, it can be seen that different equipment can be used for the presurgery inspection. According to the survey data, 69 people chose CT, 64 cases were detected, and the effective rate was 93%; 35 people chose endoscopy, 27 cases were detected, and the effective rate was 75%, 9 people chose ultrasound, and 6 cases were detected with an effective rate of 64%; 15 people chose endoscopic ultrasonography, 14 cases were detected, and the effective rate was 99%; and 20 people chose MRI, 20 cases were detected, and the effective rate was 100%. According to the survey data, the effectiveness of different equipment is different. Among them, MRI has the highest effective rate without error, followed by ultrasound endoscopy. Ultrasound has the lowest effective rate, but the effective rate also exceeds 50%. In summary, each instrument and equipment has a certain effect.

## 4. Clinical Research Based on Smart Medicine in Gastrointestinal Surgery

### 4.1. Blood Glucose Analysis

In the current medical technology, surgery is the best way to treat gastrointestinal diseases. However, different situations may vary from person to person in the field of surgery. For example, the injection of anesthetics before the operation is not risky on an objective level, but some patients will have a strong stress response, causing problems with their own immune system, which is very detrimental to the recovery of gastrointestinal patients after surgery. Therefore, the postoperative recovery of gastrointestinal surgery has also become the focus of investigation.

According to the data in Figure 6, the experiment set up an experimental group and a control group to explore the relationship between the serum and the patient's immune system. According to the serum data in the left of Figure 6, the serum should first rise and then fall after gastrointestinal surgery, and the rise is small in the early stage, and the rise is larger in the later stage. After experiencing a large increase, the serum will show a downward trend. According to the left of Figure 6, under normal conditions, the serum will experience a large degree after A2 time. A3 is the turning point of serum concentration, and there will be a subsequent decline. According to the data of the control group, it is found that the increase and decrease in the experimental group are similar, and there is no abnormality on the whole, but the specific data of the serum are indeed very different. The control group and the experimental group were not significantly different in the initial period, but the serum value began to exceed the control group at A2, and it was far beyond the normal level at A3. Although there is a downward trend after A3, the serum value is still much higher than the normal level. According to the data, the serum concentration of postoperative patients with abnormal reactions should be controlled.

The article "Clinical Research on Gastrointestinal Surgery Based on Smart Medicine" was retracted in 2022. Reason: concerns about the peer review.

According to the insulin data in the right of Figure 6, the experimental group and the control group are also set up to explore the postoperative insulin situation of patients. According to the data of the control group, the insulin of the control group experienced a trend of first rising and then falling. A3 is the turning point of insulin levels. A3 reaches the highest point of insulin, and then, there will be a sharp decline, and then, it will stabilize. According to the data of the experimental group, the overall trend of postoperative patients is not significantly different from that of the control group, but the insulin data at the same time period are far different. In the A2 time period, the insulin level has exceeded the normal level, and after the A2 time period, it has experienced a sharp rise, resulting in an abnormal situation in the insulin level. Although insulin showed a downward trend after A3, it was still in an abnormal state compared with the data of the control group. According to these data, it is known that gastrointestinal patients need to control their insulin levels after surgery to prevent abnormalities from affecting their recovery after surgery.

### 4.2. Thromboplastin Analysis

According to the data in Figure 7, to explore the postoperative insulin function changes in gastrointestinal patients, the experimental group and the control group were set up for comparison. According to the insulin function evaluation data in the left of Figure 7, the insulin function of the control group showed a trend of first rising and then falling, and the insulin function began to recover on the first day after the operation. The recovery effect is very slow at first, but there will be a sharp rise in the A2 time period, and it will reach the peak at the A3 time point. After the A3 time period, the insulin function will show a downward trend, and the downward trend will be larger at first. After the A4 time period, the decline in insulin function will be smaller and gradually maintain a stable state. From the insulin function data of the experimental group, it can be seen that, on the whole, the time points of the increase and decrease in insulin function are similar to those of the control group. However, there is a big difference in specific values, and the initial values of the experimental group and the control group are not significantly different. However, in the A2 time period, the insulin function of the experimental group far exceeded the normal level and maintained a substantial upward trend. The insulin level of the experimental group reached its peak during the A3 time period, and the insulin level at this moment was far above the normal level, which had a great impact on the patient's postoperative recovery. Although the insulin function of the experimental group showed a downward trend after the A3 time period, it was still much higher than the normal level. According to these data, it can be seen that the postoperative insulin function of gastrointestinal patients is an object that needs to be paid attention to.

The article "Clinical Research on Gastrointestinal Surgery Based on Smart Medicine" was retracted in 2022. Reason: concerns about the peer review.

According to the thromboplastin data in the right of Figure 7, the experimental group and the control group are also set up to explore the thromboplastin situation of patients after surgery. According to the data of the control group, under normal circumstances, thromboplastin will first drop and then rise after surgery. The function of thromboplastin will remain relatively stable on the first day after surgery. After the A2 period of time, thromboplastin will decrease significantly. This type of situation will remain for a period of time until A3, A3 will reach the lowest point, and then there will be an upward trend, the rise of thromboplastin will show a slow rise and a sharp rise, and it will remain stable after reaching the normal point. According to the data of the experimental group, although the characteristics of thromboplastin of gastrointestinal patients are similar to those of the control group in terms of overall trends, the specific values are quite different. There was no difference in the thromboplastin between the two in the initial period, but the thromboplastin began to decrease in a significant range from the first day after the operation, and this decline has a tendency to increase until the thromboplastin drops to the lowest point at A3. After A3, thromboplastin will show an upward trend, but the overall level is still lower than normal. According to the data, it can be known that thromboplastin in gastrointestinal patients after surgery is an object that needs to be paid attention to.

### 4.3. Serum Analysis

Serum refers to the plasma separated after blood coagulation. Serum is a complex mixture of substances. Serum will show different characteristics due to different genders, ages, and other reasons. At the same time, serum can protect cells in the body.

According to the data in Figure 8, to explore the postoperative serum changes in gastrointestinal patients, the experimental group and the control group were set up for comparison. According to the data of the left control group in Figure 8, under normal circumstances, the serum will first rise and then fall. From the first day after the operation, the serum begins to rise until it reaches the highest value at the A3 time point. After the A3 point, there will be a downward trend, and the decline will gradually become smaller, after which the serum will remain stable. From the data of the experimental group, we can see that the overall upward and downward trends are consistent with those of the control group, but the specific data are quite different. From the first day after surgery, it has increased in a larger trend. Moreover, the increase has a tendency to increase, and it seems that it will decrease in the future, but its value is still far higher than the normal level. According to the data, the postoperative serum condition of gastrointestinal patients is the object of attention.

The article "Clinical Research on Gastrointestinal Surgery Based on Smart Medicine" was retracted in 2022. Reason: concerns about the peer review.

According to the situation of the right plasma in Figure 8, under normal circumstances, the plasma will first decline and then rise, and the amplitude will continue to increase during the decline, until it reaches the lowest point, and then slowly rises to remain stable. From the data of the experimental group, it can be seen that the plasma decline trend is too large, resulting in the later plasma that cannot recover normally, and it is still in a low state. According to the data, the postoperative plasma condition of gastrointestinal patients is the object that needs to be paid attention to.

It can be seen from Figure 9 that different types of comparisons are made when analyzing plasma. Under normal circumstances, glutathione will experience a first decline and then a slow rise trend after surgery, but there will be no particularly large changes in the overall situation. However, according to the data of the experimental group, there are two different conditions for glutathione in patients after gastrointestinal surgery. The first one is a sharp decline and then rises, but this situation will cause the plasma content to be too low, which is not conducive to postoperative recovery. The second situation is that it first rises and then falls. This situation will cause the patient's postoperative plasma concentration to be too high, which is also not conducive to postoperative recovery. According to these data, we can know what kind of situation should be paid attention to when interfering with plasma condition after operation to avoid causing undesirable situations.

## 5. Conclusions

With the continuous development of society, people will pay more and more attention to health, and the shortage of medical resources will become inevitable. How to improve resource utilization and alleviate contradictions is the focus of current research. This article aims to study the clinical research of gastrointestinal surgery based on smart medicine and hopes to use smart medical technology to improve the clinical research level of gastrointestinal surgery, provide technical support for surgery, and relieve the pressure of medical workers. Although this article has carried out experimental exploration, there are still many shortcomings: (1) intelligent medical technology can summarize and categorize the medical records of doctors. However, due to the differences in the personal experience and abilities of doctors, there will be differences when writing medical records. There is not much discussion in this part. (2) The postoperative complications of gastrointestinal patients have not been explored too much.

The article "Clinical Research on Gastrointestinal Surgery Based on Smart Medicine" was retracted in 2022. Reason: concerns about the peer review.

## Figures and Tables

**Figure 1:** Original smart medical structure.

**Figure 2:** Wearable smart health care.

**Figure 3:** Intelligent diagnostic system.

**Figure 4:** Schematic diagram of the sample.

**Figure 5:** Whole process of surgery.

**Figure 6:** Comparative analysis of blood glucose and insulin.

**Figure 7:** Functional evaluation and thromboplastin analysis.

**Figure 8:** Serum and plasma analysis.

**Figure 9:** Comparative analysis of plasma levels.

**Table 1:** Age distribution of patients.

Age (years)	Male	Ratio (%)	Female	Ratio (%)
0–20	2	1.3	1	0.7
21–40	17	11.4	13	8.8
41–60	25	16.9	19	12.9
60–80	39	26.6	32	21.7
Total	83	56.1	65	43.9

**Table 2:** Clinical manifestations of gastrointestinal disease.

Manifestations	Number	Proportion (%)
Gastrointestinal bleeding	27	18
Difficulty swallowing	10	7
Abdominal pain and distention	78	53
Black stools	19	13
Other	14	9
Total	148	100

**Table 3:** Investigation of gastrointestinal disease site.

Part	Number	Proportion (%)
Ovary	3	2
Colorectum	19	13
Peritoneum	7	5
Uterus	2	1
Stomach	96	65
Duodenum	21	14
Total	148	100

**Table 4:** Preoperative examination of patients.

Category	Number of detections	Total number	Effective percentage
CT	64	69	93
Endoscopy	27	35	75
Ultrasound	6	9	64
Ultrasound endoscopy	14	15	99
MRI	20	20	100
Total	131	148	88.5

## Data Availability

No data were used to support this study.
